# The Nuclear Orphan Receptor Nur77 Alleviates Palmitate-induced Fat Accumulation by Down-regulating G0S2 in HepG2 Cells

**DOI:** 10.1038/s41598-018-23141-8

**Published:** 2018-03-19

**Authors:** Naiqian Zhao, Xiaoyan Li, Ying Feng, Jinxiang Han, Ziling Feng, Xifeng Li, Yanfang Wen

**Affiliations:** 1 Department of Gerontology, Second Hospital of Shanxi Medical University, 382 Wuyi Road, Taiyuan, 030001 Shanxi China; 2 Department of Infectious Diseases, First People’s Hospital of Jinzhong, 85 Shuncheng Street, Jinzhong, 030600 Shanxi China

## Abstract

Excessive triglyceride accumulation in hepatocytes is the hallmark of obesity-associated nonalcoholic fatty liver disease (NAFLD). Elevated levels of the saturated free fatty acid palmitate in obesity are a major contributor to excessive hepatic lipid accumulation. The nuclear orphan receptor Nur77 is a transcriptional regulator and a lipotoxicity sensor. Using human HepG2 hepatoma cells, this study aimed to investigate the functional role of Nur77 in palmitate-induced hepatic steatosis. The results revealed that palmitate significantly induced lipid accumulation and suppressed lipolysis in hepatocytes. In addition, palmitate significantly suppressed Nur77 expression and stimulated the expression of peroxisome proliferator-activated receptor γ (PPARγ) and its target genes. Nur77 overexpression significantly reduced palmitate-induced expression of PPARγ and its target genes. Moreover, Nur77 overexpression attenuated lipid accumulation and augmented lipolysis in palmitate-treated hepatocytes. Importantly, G0S2 knockdown significantly attenuated lipid accumulation and augmented lipolysis in palmitate-treated hepatocytes, whereas G0S2 knockdown had no effect on the palmitate-induced expression of Nur77, PPARγ, or PPARγ target genes. In summary, palmitate suppresses Nur77 expression in HepG2 cells, and Nur77 overexpression alleviates palmitate-induced hepatic fat accumulation by down-regulating G0S2. These results display a novel molecular mechanism linking Nur77-regulated G0S2 expression to palmitate-induced hepatic steatosis.

## Introduction

Obesity is increasing at an explosive rate worldwide due to an increase in total energy consumption and a shift in the types of nutrients consumed^1,2^. The pandemic rise in obesity has resulted in an increased incidence of obesity-associated nonalcoholic fatty liver disease (NAFLD)^3^. Consequently, NAFLD has become an emerging public health problem and is now the most common cause of chronic liver disease in much of the world^4,5^. Obesity is associated with increased circulating levels of nonesterified or free fatty acids (FFAs), compounds that are taken up by the liver, where they are esterified into neutral triglycerides^6^. An increased supply of FFAs to the liver results in excessive accumulation of neutral triglyceride droplets within hepatocytes, which is the hallmark of NAFLD^7^. Prior studies have demonstrated that the saturated fatty acid palmitate, which makes up 30–40% of high plasma FFA concentrations^8^, contributes to the accumulation of excess triglycerides in hepatocytes^9,10^. However, the molecular mechanism connecting palmitate to NAFLD has not been fully elucidated.

A decreased rate of triglyceride mobilization plays a key role in triglyceride accumulation in the liver^11,12^. The cleavage of the first ester bond in triglycerides, which is catalysed by adipose triglyceride lipase (ATGL)13, is the rate-limiting step in intracellular triglyceride hydrolysis, and ATGL activity is governed by several regulatory proteins^13,14^. Specifically, the protein product encoded by G0/G1 switch gene 2 (G0S2) is a dominant specific inhibitor of ATGL^15^. G0S2 binds directly to ATGL and attenuates ATGL-mediated lipolysis by inhibiting the triglyceride hydrolase activity of ATGL in adipose tissue and other tissues^14–16^. G0S2 was recently shown to be a major contributor to the development of hepatic steatosis^17,18^. Moreover, *in vitro* and *in vivo* studies have demonstrated that G0S2 is a direct target gene of peroxisome proliferator-activated receptor γ (PPARγ), and the activation of PPARγ can up-regulate G0S2 expression^19^.

The nuclear orphan receptor NR4A subfamily belongs to the nuclear hormone receptor superfamily and contains three members, namely, NR4A1, NR4A2, and NR4A3, which are also known as Nur77, Nurr1, and Nor1, respectively^20^. Of the NR4A members, Nur77 shows the most widespread tissue distribution and is mainly expressed in metabolically demanding and energy-dependent tissues^21^. Nur77 affects gluconeogenesis and lipogenesis in the liver and energy expenditure in brown adipose tissue and possibly white adipose tissue (WAT)^22–25^. Nur77 deletion leads to hepatic steatosis in high fat-fed mice, which suggests that Nur77 contributes to excess triglyceride accumulation in hepatocytes^24^. Interestingly, Nur77 expression is significantly induced in WAT during fasting, whereas PPARγ expression is significantly decreased, which implies that Nur77 might inhibit PPARγ expression^25^. Additionally, in mature 3T3-L1 adipocytes that are serum starved in a low-glucose medium, stimulation with the β-adrenergic agonist isoprenaline rapidly increases the mRNA expression of Nur77 and decreases the PPARγ expression level decreases, confirming that the overexpression of Nur77 suppresses PPARγ expression under various metabolic conditions^25^. In Nur77^−/−^ mice, PPARγ expression in WAT depots is significantly up-regulated, and this up-regulation of PPARγ is also reflected by an increased expression of a known downstream target gene of PPARγ, G0S2^25^. Further chromatin immunoprecipitation and luciferase assays have shown that Nur77 directly binds to and represses the PPARγ promoter and reduces the expression of PPARγ and PPARγ-regulated downstream target genes^25^. These findings demonstrate that Nur77 is a direct repressor of PPARγ expression.

Based on these observations, we made the following hypothesis: (1) palmitate suppresses Nur77 and subsequently stimulates the expression of its downstream target PPARγ and G0S2, (2) this increase in G0S2 expression contributes to palmitate-induced fat accumulation in the liver, and (3) Nur77 overexpression suppresses G0S2 expression in the liver, thereby exerting a protective effect against palmitate-induced hepatic steatosis. In this study, we examined the functional involvement of Nur77, PPARγ, and G0S2 in HepG2 hepatocytes treated with palmitate. HepG2 cells have been extensively used as a cellular model for research on hepatic steatosis^26^. We analysed the expression patterns of the aforementioned proteins and performed both gain- and loss-of-function experiments via plasmid-mediated protein overexpression and small interfering RNA (siRNA)-mediated gene knockdown. Our results provide novel information regarding the molecular mechanism through which palmitate induces fat accumulation in hepatocytes.

## Results

### Palmitate induced lipid accumulation and suppressed lipolysis in HepG2 cells

HepG2 cells were incubated with increasing concentrations of palmitate for 24 h, and the resulting intracellular accumulation of lipids was examined through Oil Red O staining. Consistent with a previous report^10^, palmitate caused a dose-dependent increase in lipid accumulation in HepG2 cells (Fig. 1A and B). Moreover, the incubation of HepG2 cells with palmitate also decreased lipolysis in a dose-dependent manner, as demonstrated by reductions in the release of glycerol into the media (Fig. 1C). Palmitate at a concentration of 200 μM, which represents a high physiological level in the circulation of obese individuals^27^, induced a significant increase in lipid accumulation and a significant decrease in lipolysis. Therefore, this concentration of palmitate was used in all the following plasmid overexpression and siRNA knockdown experiments.

**Figure 1:** Palmitate induced lipid accumulation and suppressed lipolysis in HepG2 cells. (**A** and **B**) Dose–response relationship between palmitate and lipid accumulation. (**A**) HepG2 cells were stained with Oil Red O to visualize the intracellular lipid contents (original magnification, ×100). (**B**) Lipid accumulation was quantified by the absorbance value of the extracted Oil Red O dye at 500 nm. The data from each group are presented as the means ± SEs (n = 3). **P < 0.01. (**C**) Dose–response relationship between palmitate and inhibition of lipolysis. Lipolysis was assessed by the release of glycerol into the media. The data from each group are presented as the means ± SEs (n = 3). **P < 0.01.

### Palmitate suppressed Nur77 expression and stimulated expression of PPARγ and its target genes in HepG2 cells

As shown in previous studies, the transcription factors Nur77 and PPARγ are involved in hepatic lipid accumulation^9,24^. To elucidate the molecular mechanism of palmitate-induced hepatic lipid accumulation, we examined the effects of palmitate on the expression of Nur77, PPARγ, and several known PPARγ target genes in HepG2 cells. HepG2 cells were incubated with increasing concentrations of palmitate for 24 h, and a quantitative PCR analysis revealed that palmitate induced a dose-dependent decrease in Nur77 mRNA expression and a dose-dependent increase in the mRNA expression of PPARγ and its target genes (G0S2, GPR81, GPR109A, and Adipoq) (Fig. 2A). Additionally, a Western blot analysis showed that the incubation of HepG2 cells with palmitate yielded a dose-dependent decrease in Nur77 protein expression and a dose-dependent increase in PPARγ and G0S2 protein expression (Fig. 2B).

**Figure 2:** Palmitate suppressed Nur77 expression and stimulated the expression of PPARγ and its target genes in HepG2 cells. (**A**) Palmitate suppressed Nur77 mRNA expression and stimulated the mRNA expression of PPARγ and its target genes (G0S2, GPR81, GPR109A, and Adipoq) in a dose-dependent manner. The mRNA levels were measured by a quantitative PCR analysis. The data from each group are presented as the means ± SEs (n = 3). *P < 0.05, **P < 0.01. (**B**) Palmitate suppressed Nur77 protein expression and stimulated PPARγ and G0S2 protein expression in a dose-dependent manner. Protein expression was examined through a Western blot analysis. The data from each group are presented as the means ± SEs (n = 3). **P < 0.01.

### Nur77 suppressed the expression of palmitate-induced PPARγ and its target genes in HepG2 cells

We subsequently examined whether Nur77 regulates the palmitate-induced expression of PPARγ and its target genes in HepG2 cells. HepG2 cells were transfected with pReceiver-M98-Nur77 to overexpress Nur77 and then treated with 200 μM palmitate for 24 h. As shown in Fig. 3A, pReceiver-M98-Nur77 transfection efficiently increased Nur77 protein expression. A quantitative PCR analysis revealed that Nur77 overexpression significantly decreased the palmitate-induced mRNA expression of PPARγ and its target genes (G0S2, GPR81, GPR109A, and Adipoq) (Fig. 3B). Additionally, a Western blot analysis showed that Nur77 overexpression significantly decreased palmitate-induced PPARγ and G0S2 protein expression (Fig. 3C).

**Figure 3:** Nur77 suppressed the palmitate-induced expression of PPARγ and its target genes in HepG2 cells. (**A**) HepG2 cells were transfected with pReceiver-M98 or pReceiver-M98-Nur77, and Nur77 expression was measured through a Western blot analysis. The data from each group are presented as the means ± SEs (n = 3). **P < 0.01. (**B**) Nur77 overexpression decreased the palmitate-induced mRNA expression of PPARγ and its target genes (G0S2, GPR81, GPR109A, and Adipoq). mRNA expression was measured by a quantitative PCR analysis. The data from each group are presented as the means ± SEs (n = 3). *P < 0.05, **P < 0.01. (**C**) Nur77 overexpression decreased the palmitate-induced protein expression of PPARγ and G0S2. Protein expression was measured through a Western blot analysis. The data from each group are presented as the means ± SEs (n = 3). **P < 0.01.

### Nur77 attenuated lipid accumulation and augmented lipolysis in palmitate-treated HepG2 cells

Because Nur77 has been associated with hepatic steatosis^24^, we also investigated the effects of Nur77 on lipid accumulation and lipolysis in palmitate-treated HepG2 cells. HepG2 cells were transfected with pReceiver-M98-Nur77 and then treated with 200 μM palmitate for 24 h. As shown in Fig. 4A, Nur77 overexpression significantly attenuated palmitate-induced lipid accumulation in HepG2 cells. In addition, Nur77 overexpression significantly augmented lipolysis in palmitate-treated HepG2 cells (Fig. 4B).

**Figure 4:** Nur77 attenuated lipid accumulation and augmented lipolysis in palmitate-treated HepG2 cells. (**A**) Nur77 overexpression decreased palmitate-induced lipid accumulation. Lipid accumulation was detected through Oil Red O staining and quantified by the absorbance of the extracted Oil Red O dye at 500 nm. The data from each group are presented as the means ± SEs (n = 3). **P < 0.01. (**B**) Nur77 overexpression increased lipolysis in palmitate-treated HepG2 cells. Lipolysis was assessed by the release of glycerol into the media. The data from each group are presented as the means ± SEs (n = 3). *P < 0.05.

### G0S2 knockdown attenuated lipid accumulation and augmented lipolysis in palmitate-treated HepG2 cells

G0S2 is a key contributor to the development of fatty liver^17,18^. We therefore studied the effects of G0S2 on lipid accumulation and lipolysis in palmitate-treated HepG2 cells. HepG2 cells were transfected with G0S2 siRNA and then treated with 200 μM palmitate for 24 h. G0S2 siRNA efficiently decreased G0S2 protein expression (Fig. 5A), and G0S2 knockdown significantly attenuated palmitate-induced lipid accumulation in HepG2 cells (Fig. 5B). In addition, G0S2 knockdown significantly augmented lipolysis in palmitate-treated HepG2 cells (Fig. 5C). However, G0S2 knockdown had no effect on the mRNA expression of Nur77, PPARγ, or the PPARγ target genes of interest (GPR81, GPR109A, and Adipoq) (Fig. 5D) or on the protein expression of Nur77 or PPARγ in palmitate-treated HepG2 cells (Fig. 5E).

**Figure 5:** G0S2 knockdown attenuated lipid accumulation and augmented lipolysis in palmitate-treated HepG2 cells. (**A**) HepG2 cells were transfected with control siRNA or G0S2 siRNA, and G0S2 expression was measured through a Western blot analysis. The data from each group are presented as the means ± SEs (n = 3). **P < 0.01. (**B**) G0S2 knockdown decreased palmitate-induced lipid accumulation. Lipid accumulation was detected through Oil Red O staining and quantified by the absorbance of the extracted Oil Red O dye at 500 nm. The data from each group are presented as the means ± SEs (n = 3). *P < 0.05. (**C**) G0S2 knockdown increased lipolysis in palmitate-treated HepG2 cells. Lipolysis was assessed by the release of glycerol into the media. The data from each group are presented as the means ± SEs (n = 3). *P < 0.05. (**D**) G0S2 knockdown did not affect the mRNA expression of Nur77, PPARγ, or the PPARγ target genes of interest (GPR81, GPR109A, and Adipoq). mRNA expression was measured through quantitative PCR analysis. The data from each group are presented as the means ± SEs (n = 3). (**E**) G0S2 knockdown did not affect Nur77 or PPARγ protein expression. Protein expression was measured through a Western blot analysis. The data from each group are presented as the means ± SEs (n = 3).

## Discussion

In obese individuals, elevated plasma FFA levels, which are due to accelerated FFA release rates under basal^28^ and postprandial^29^ conditions, cause excess lipid accumulation in nonadipose tissues. Elevated plasma levels of palmitate, which is the most abundant saturated fatty acid in plasma^30^, play an aetiological role in the development of NAFLD and are postulated to constitute a critical link between obesity and the risk of NAFLD^31^. Several studies have demonstrated that palmitate induces lipid accumulation in HepG2 cells^10,32^. In this study, we once again confirmed that palmitate induces intracellular lipid accumulation and suppresses lipolysis in hepatocytes.

In recent years, the nuclear orphan receptor Nur77 has been implicated in metabolic regulation via actions in the liver, skeletal muscle, and adipose tissue^33^. Nur77 expression is known to be induced by a diverse range of signals, including oxidative stress, growth factors, cytokines, and lipotoxic fatty acids, and alterations in its expression can regulate its transcriptional activity^34^. Several studies have shown that Nur77 plays a direct role in gene regulation during the fasting responses of several major metabolic tissues^25^. Specifically, in fasting WAT, Nur77 expression is significantly induced, and PPARγ expression is significantly decreased^25^. Chromatin immunoprecipitation and luciferase assays have shown that Nur77 directly binds to and represses the PPARγ promoter, which implies that changes in PPARγ expression are responsible for the metabolic regulatory functions of Nur77^25^. PPARγ plays a pivotal role and is absolutely necessary in adipogenesis^35^. By regulating the expression of many target genes, this molecule influences the recycling of intracellular fatty acids, promoting lipid storage and lipogenesis. G0S2, GPR81, GPR109A, and Adipoq are known downstream target genes of PPARγ that are involved in lipolysis under distinct physiological conditions^25,36^. Several studies have demonstrated that Nur77 overexpression is capable of blocking adipogenesis in adipocytes^37,38^. In particular, a quantitative analysis of the liver lipid content has confirmed that the liver tissue of Nur77-null mice accumulates more triglycerides than that of wild-type mice, reflecting the beneficial effect of Nur77 on hepatic steatosis^24^. However, the functional role of Nur77 in palmitate-induced hepatic lipid accumulation remains unknown. In this study, we found that palmitate causes dose-dependent decreases in Nur77 mRNA and protein expression and dose-dependent increases in the mRNA expression of PPARγ and its target genes (G0S2, GPR81, GPR109A, and Adipoq) and the protein expression of PPARγ and G0S2 in HepG2 cells. We also found that Nur77 overexpression significantly decreased the mRNA expression levels of PPARγ and its target genes (G0S2, GPR81, GPR109A, and Adipoq) and the protein expression of PPARγ and G0S2 in palmitate-treated HepG2 cells. In addition, Nur77 overexpression attenuated lipid accumulation and augmented lipolysis in palmitate-treated HepG2 cells. These findings suggested that the down-regulation of PPARγ and its lipolysis-related target genes by Nur77 might be an important mechanism for alleviating palmitate-induced excessive lipid accumulation in hepatocytes.

The aforementioned PPARγ target genes are involved in lipolysis under varying metabolic conditions. During fasting, G0S2 expression increases in the liver and decreases in adipose tissue^17^. G0S2 knockout notably decreases the hepatic triglyceride content, whereas G0S2 overexpression induces triglyceride accumulation and promotes fatty liver formation^17,18^. G protein-coupled receptor 81 (GPR81) has been identified as a specific receptor for lactate and mediates the insulin-dependent inhibition of lipolysis through both autocrine and paracrine actions^36,39^. G protein-coupled receptor 109A (GPR109A) functions as a receptor for the ketone body 3-hydroxybutyric acid and is a metabolic sensor that mediates antilipolytic actions during starvation to avoid excessive triglyceride degradation^40,41^. Adiponectin (encoded by Adipoq) is a adipokine that can augment the oxidation of fatty acids to alleviate hepatic lipid accumulation^42^. However, Adipoq is down-regulated in obesity^43^. Therefore, G0S2 might play a critical role in Nur77-regulated hepatic lipid accumulation. A recent study showed that fatty acids derived from adipose tissue up-regulate fasting G0S2 expression in the liver to induce hepatic triglyceride accumulation^44^. However, the contribution of G0S2 to palmitate-induced hepatic lipid accumulation has not been previously explored. In this study, we found that G0S2 knockdown significantly attenuated lipid accumulation and augmented lipolysis in palmitate-treated HepG2 cells. More importantly, the inhibition of G0S2 expression had no effect on the mRNA expression of Nur77, PPARγ, or the PPARγ target genes examined (GPR81, GPR109A, and Adipoq) or on the protein expression of Nur77 or PPARγ in palmitate-treated HepG2 cells. Together, these results indicate that palmitate suppresses Nur77 expression in HepG2 cells and that Nur77 overexpression alleviates palmitate-induced hepatic fat accumulation by down-regulating G0S2. Based on these findings, we speculate that decreased Nur77 expression in palmitate-induced hepatic steatosis, coupled with increased G0S2 expression, represents a molecular mechanism connecting palmitate to NAFLD, which strengthens the emerging potential of Nur77 as a candidate for the treatment of obesity-associated NAFLD. However, in pancreatic β-cells, palmitate induces Nur77 expression^45^, indicating that palmitate regulates Nur77 expression in a tissue-dependent manner, and the target genes and functions of Nur77 are likely tissue-dependent. Thus, the extrapolation of Nur77 gene expression data to a pharmacological intervention strategy needs to be carefully considered. Further investigations are needed to address the tissue-specific gene expression profiles and functions of Nur77.

## Methods

### Cell culture

HepG2 cells, a human hepatoma cell line (China Center for Type Culture Collection, Wuhan, China), were maintained in Dulbecco’s modified Eagle’s medium (DMEM; Invitrogen, Carlsbad, CA, USA) containing 10% foetal bovine serum (FBS; Invitrogen), 100 U/mL penicillin, 100 µg/mL streptomycin, and 1% L-glutamine. The cells were cultured in cell culture flasks at 37 °C in a humidified atmosphere containing 5% CO_2_ and 95% air. The effect of palmitate was examined by the addition of this agent to cells plated in six-well plates at 2 × 10^5^ cells/well.

### Preparation of palmitate solution

A palmitate (Sigma, St. Louis, MO, USA) stock solution was prepared by coupling palmitate to bovine serum albumin (BSA; Sigma) as previously described^46^. Briefly, palmitate was fully dissolved in 100% ethanol to obtain a concentration of 195 mM, and the final concentration of ethanol in the palmitate stock solution did not exceed 1.5% by volume. The prepared palmitate stock solution was then mixed with a prewarmed BSA solution (10% w/w, 37 °C) to allow palmitate to bind to albumin and achieve a final palmitate concentration of 3 mM. Palmitate was fully dissolved by incubating the mixture in a water bath at 37 °C for 10 min. The final molar ratio of palmitate to BSA was 2:1. The control vehicle was prepared using a stock of 10% w/w BSA with an equivalent volume of ethanol to match that contained in the final palmitate stock. The final concentration of ethanol was less than 0.2% by volume in all the experiments.

### Quantitative real-time PCR analysis

The Total RNA from cultured HepG2 cells was isolated using the TRIzol^®^ reagent (Invitrogen) according to the manufacturer’s instructions. The RNA concentration and quality were evaluated with a Nanodrop ND1000 spectrophotometer (Thermo Scientific, Wilmington, DE, USA). The Total RNA (500 ng) was used for reverse transcription (RT) using SuperScript II reverse transcriptase (Invitrogen). The RT conditions for each cDNA amplification were 42 °C for 15 min, 85 °C for 5 s, and 4 °C for ∞, and the products were stored at −20 °C. For the quantification of gene expression, quantitative PCR (qPCR) was performed with a StepOnePlus^TM^ Real-Time PCR System (Applied Biosystems, Inc., Foster City, CA, USA) using SYBR Green as the detection dye. The primer sequences designed for gene detection were as follows: Nur77 forward primer, 5′-CTGCCCTTGTCCTCATCACC-3′; reverse primer, 5′- CAGTTTGCCCAACAGACGT-3′; PPARγ forward primer, 5′-ACCACTCCCACTCCTTTG-3′; reverse primer, 5′-GCAGGCTCCACTTTGATT-3′; G0S2 forward primer, 5′-CCTCTTCGGCGTGGTGCT-3′; reverse primer, 5′-CTGCTGCTTGCCTTTCTCC-3′; GPR81 forward primer, 5′-CAGACAGGCTCGGATGAAGAAG-3′; reverse primer, 5′-TTGTAGAATTTGGGAAAGGAGGG-3′; GPR109A forward primer, 5′-TGGACCTGGCGTTCTTTA-3′; reverse primer, 5′-GCTCGTGCTGCGGTTATT-3′; Adipoq forward primer, 5′-AGGAAAGGAGAACCTGGAGAAG-3′; reverse primer, 5′- ATAGACTGTGATGTGGTAGGCAAA-3′; β-actin forward primer, 5′-TGGCACCCAGCACAATGAA-3′; and reverse primer, 5′-CTAAGTCATAGTCCGCCTAGAA-3′. The expected lengths of the amplified product were 158 bp (Nur77), 169 bp (PPARγ), 160 bp (G0S2), 240 bp (GPR81), 170 bp (GPR109A), 204 bp (Adipoq) and 186 bp (β-actin). β-Actin was used as the control housekeeping gene. The cycling conditions consisted of 45 cycles of 94 °C for 5 s and 60 °C for 30 s. The predicted length of the PCR product was identified by 2% agarose gel electrophoresis with ethidium bromide staining. To monitor the specificity of the amplified PCR product, we performed a melting curve analysis for each sample in direct connection to the PCR assay. The results were analysed using the 2^−ΔΔCt^ method and are presented as the fold differences in the expression of each target gene compared to that of β-actin in the same sample. All the samples were processed in duplicate.

### Western blot analysis

The HepG2 cells were harvested and lysed with ice-cold RIPA lysis buffer containing protease inhibitor cocktail (Roche Diagnostics, Mannheim, Germany). The protein concentration was determined using a Bio-Rad DC protein assay kit (Bio-Rad, Hercules, CA, USA) according to the manufacturer’s instructions. Briefly, after boiling to achieve protein denaturation, equal amounts of total protein (40 µg) were loaded onto gels and resolved by 10% sodium dodecyl sulphate polyacrylamide gel electrophoresis (SDS-PAGE) for 2 h at room temperature. The proteins were subsequently transferred to polyvinylidene difluoride (PVDF) membranes (Atto Corporation, Tokyo, Japan). The membranes were blocked with 5% non-fat milk dissolved in TBS-T buffer for 2 h and probed first with primary antibodies overnight and then with secondary antibodies for 1 h. The primary antibodies used were anti-Nur77 (1:200, Santa Cruz Biotechnology, Santa Cruz, CA, USA), anti-PPARγ (1:1000, Cell Signalling, NEB, Vienna, Austria) and anti-G0S2 (1:100, Sigma). An anti-β-actin antibody (1:2000, Sigma) was used as the loading control. The secondary antibody was goat anti-rabbit IgG-horseradish peroxidase conjugate (1:2000, Bio-Rad). The immunoreactive protein bands were visualized using an enhanced chemiluminescence (ECL) detection system (Amersham Pharmacia Biotech, Piscataway, NJ, USA) according to the manufacturer’s instructions. The density of the band was determined using ImageJ software (NIH, Bethesda, MD, USA), and the data were transformed and normalized relative to β-actin to obtain the integral optical density (IOD) ratio. All the experiments were performed at least three times, and representative data are shown.

### siRNA-mediated knockdown

For the siRNA experiments, an RNA oligonucleotide directed against G0S2 (sense sequence: GCATCCACCAAAGGAGTTTGG) for silencing the target gene and a negative control siRNA with no matches in the human genome were also purchased from GeneChem Co., Ltd. (Shanghai, China). HepH2 cells were transfected with these siRNAs using Lipofectamine 2000 (Invitrogen) according to the manufacturer’s instructions. Briefly, HepG2 cells were seeded into six-well plates and cultured overnight. The aforementioned siRNAs (2.5 µg of each) and 5 μL of Lipofectamine^®^ 2000 reagent were diluted in 250 µL of Opti-MEM^®^ medium (Invitrogen) and incubated separately for 10 min at room temperature. After the 10-min incubation, equal volumes of the diluted siRNA and Lipofectamine^®^ 2000 reagent were mixed gently, and the mixtures were incubated for 10 min at room temperature to form siRNA-lipid complexes. For transfection, the siRNA-lipid complexes were subsequently combined with HepG2 cells in six-well culture plates at 1 × 10^6^ cells/well and incubated for 24 h. The knockdown efficiency of the siRNAs was determined by Western blot analysis. The transfected cells were then treated with 200 μM palmitate for 24 h and harvested.

### Plasmid-mediated overexpression

The pReceiver-M98-Nur77 and pReceiver-M98 plasmids were purchased from GeneCopoeia Inc. (Guangzhou, China). The pReceiver-M98 plasmid was used as a control. The plasmid transfection experiments were performed using Lipofectamine 2000 (Invitrogen) according to the manufacturer’s instructions. The HepG2 cells were plated at 1 × 10^5^ cells/well on six-well culture plates and cultured overnight. After the cells were washed twice with fresh DMEM, the wells were then filled with fresh DMEM (2.0 ml/well). The pReceiver-M98-Nur77 and pReceiver-M98 plasmids (2.5 μg) and 5 μL of Lipofectamine 2000 reagent were diluted in 250 μL of Opti-MEM^®^ Medium (Invitrogen) and incubated separately for 10 min at room temperature. Equal volumes of the plasmid dilution and Lipofectamine^®^ 2000 reagent were mixed gently, and the mixtures were incubated for 10 min at room temperature to form plasmid-lipid complexes. The plasmid-lipid complexes were subsequently added to each well. The cells were cultured for 24 h at 37 °C, and the medium was then replaced with fresh DMEM containing 10% FBS (2.0 mL/well). The cells were incubated for another 24 h before use. The transfection efficiency of the plasmids was detected by Western blot analysis.

### Oil Red O staining

HepG2 cells were grown on six-well plates, washed three times with phosphate-buffered saline (PBS), and fixed with 10% formaldehyde for 30 min at room temperature. The fixed cells were washed with ddH_2_O, dipped in 60% isopropanol for 3 min, and stained with 2 mg/mL Oil Red O (Sigma) staining solution for 60 min. After staining, the cells were washed three times with ddH_2_O to remove any unbound dye. The cell nuclei were counterstained with haematoxylin for 3 min and washed with ddH_2_O. Images were obtained using an Axiovert 40 CFL microscope (Olympus, Tokyo, Japan). After the microscopic examination, the amount of triglyceride in each well was determined by measuring the amount of Oil Red O. After the cells were washed and dried completely, 200 μL of isopropanol extraction solution was added to each stained well, and the mixtures were incubated for 10 min and subjected to gentle vibration for 10 min at room temperature to release the Oil Red O stain. The extracted dye was removed by gentle pipetting, and its absorbance at 500 nm was read with a microplate reader (VersaMax; Molecular Devices Corporation, CA, USA). All the tests were performed in triplicate.

### Measurement of lipolysis

Lipolysis was assessed by measuring the amount of glycerol released into the media. Aliquots of culture media were centrifuged to remove debris and directly subjected to glycerol measurement. The amounts of glycerol released were quantified using a glycerol quantification kit according to the manufacturer’s instructions (Biovision, Inc., Milpitas, CA, USA). The glycerol levels were measured by detecting the absorbance at 550 nm using an autoanalyser (Cobas-Mira; Roche Diagnostics, Basel, Switzerland) following the manufacturer’s instructions. All the samples were measured in duplicate.

### Statistical analyses

All the experimental data are presented as the means ± SEs. Statistical differences were evaluated by Student’s *t*-test or one-way analysis of variance (ANOVA) as appropriate using SPSS 18.0 analysis software (SPSS, Chicago, IL, USA). The differences were considered significant at *P* < 0.05.

### Data availability statement

All data are fully available without restriction.
